The article "Isolation, characterization and anti-inflammatory activity of compounds from the Vernonia amygdalina" was retracted in 2025. Reasons: unreliable results or conclusions; concerns about the citations; concerns about the authorship.

# Isolation, characterization and anti-inflammatory activity of compounds from the *Vernonia amygdalina*

**DOI:** 10.1016/j.heliyon.2024.e29518

**Published:** 2024-04-13

**Authors:** Olubunmi Atolani, Mohammed Abubakar Usman, Jamiu Opeyemi Adejumo, Adedamola Elizabeth Ayeni, Olamilekan Joseph Ibukun, Adeola T. Kola-Mustapha, Ngaitad S. Njinga, Luqman A. Quadri, Emmanuel O. Ajani, Tajudeen O. Amusa, Moji T. Bakare-Odunola, Adenike T. Oladiji, Athba Alqahtani, Mohamed Abbas, Learnmore Kambizi

**Affiliations:** a African Centre for Herbal Research, Ilorin (ACHRI), University of Ilorin, Nigeria; b Department of Chemistry, University of Ilorin, Ilorin, Nigeria; c Department of Chemical Sciences, Indian Institute of Science Education and Research Kolkata, Mohanpur, 741246, West Bengal, India; d Department of Pharmaceutics and Industrial Pharmacy, University of Ilorin, Ilorin, Nigeria; e Department of Pharmaceutical and Medicinal Chemistry, University of Ilorin, Ilorin, Nigeria; f Department of Biochemistry, University of Ilorin, Ilorin, Nigeria; g Phytomedicine Toxicology and Drug Development Laboratory, Department of Biochemistry, Kwara State University, Malete, Nigeria; h Department of Forest Research Management, University of Ilorin, Ilorin, Nigeria; i Research Centre, King Fahad Medical City. P.O. Box: 59046, Riyadh 11525, Saudi Arabia; j Electrical Engineering Department, College of Engineering, King Khalid University, Abha 61421, Saudi Arabia; k Department of Hulticulture, Cape Peninsula University of Technology, South Africa

**Keywords:** Bioactive, Nuclear magnetic resonance, Spectroscopy, Vernoamyoside, Glycoside

## Abstract

The need to explore the abundance of natural products cannot be overemphasized particularly in the management of various disease conditions. In traditional medical practice, *Vernonia amygdalina* has been widely adopted in the management of various inflammatory disorders. The objective of this investigation was to isolate the bioactive principles from the stem-bark and root of *V. amygdalina* and assess the anti-inflammatory (*in vitro*) activity of both the crude extracts and the isolated compounds. Following extraction with the methanol, the extract was subjected to gravity column chromatography and the resultant fractions was further purified to obtained pure compounds. The structural elucidation of the compounds were based on data obtained from 1H to 13C nuclear magnetic resonance (NMR) spectroscopies as well as fourier transform infrared (FT-IR). Using diclofenac as a control drug, the albumin denaturation assay was used to determine the *in vitro* anti-inflammatory activity of the extracts and isolates. Three distinct compounds characterized are vernoamyoside D, luteolin-7-α-o-glucuronide, and vernotolaside, a new glycoside. When compared to diclofenac, which has an IC_50_ of 167.8 μg/mL, luteolin-7-α-o-glucuronide, vernoamyoside D, and vernotolaside all showed significant inhibitions with respective IC_50_ values 549.8, 379.5, and 201.7 μg/mL. Vernotolaside is reported for the first time from the root. The assertion that the plant is used in traditional medicine for the management of inflammatory disorder is somewhat validated by the confirmation of the existence of the compounds with the biochemical actions. Further validation of the isolated compounds would be required in animal studies.

The article "Isolation, characterization and anti-inflammatory activity of compounds from the Vernonia amygdalina" was retracted in 2025. Reasons: unreliable results or conclusions; concerns about the citations; concerns about the authorship.

## 1 Introduction

*Vernonia amygdalina* of the family Asteraceae is one of the most nutritional culinary medicinal plants in primarily in the tropical regions. On the account of his bitter taste, it is often referred to as “bitter leaf” [1]. *V. amygdalina* is a perennial shrub that reaches 3 m in height in the tropics [2]. The plant is grown by some tribes who uses it for culinary purpose in Nigeria [3]. The macerated leaves of the plant are consumed as vegetables and condiments. Interestingly, the aqueous leaf extract is applied topically for wound healing [4,5]. The plant is renowned for its protective effects in various genotoxicity, cardiotoxicity and hepatotoxicity studies [[6], [7], [8]]. The crude extract of the leave is also reported to possess anti-inflammatory potential [[9], [10], [11]] and synergistic anti-cancer effects with gemcitabine [12]. The plant have many other non-medicinal applications particularly in nanoparticle preparations [13]. Bioactive principles have been obtained from various parts of plants which include the leaves, stem, wood, root, flowers and seed [14]. The root of plant has been a source isolation of bioactive principles [[15], [16], [17], [18]]. While nanoparticles have been used for various things like biosensor preparation [19,20], the nanoparticles produced from the plant exhibited anti-inflammatory and antinociceptive activities in the animal model [21,22]. In this study, we isolated and characterized the major bioactive principles from *V. amygdalina* root and stem bark. The *in vitro* anti-inflammatory potentials using albumin denaturing inhibition assay was also evaluated.

## 2 Materials and Methods

### 2.1 General

A silica gel 60F_264_ Merck, Darmstadt, Germany precoated TLC plates (0.2 mm layer thickness) was used for spotting and visualisation carried out under short and long wavelengths of the UV-lamp or by reaction of the developed plate with iodine vapour in the iodine chamber for 1 min. Fractionation was performed on silica gel-loaded column chromatography (CC). For the determination of the functional groups in the isolated compound, a Shimadzu (8400s) Fourier Transform-Infrared (FT-IR), Shimadzu, Japan, was used to generate the infrared spectra using potassium bromide pellets. ^1^H and ^13^C NMR spectra were obtained in chloroform-*d*_*3*_ on Bruker 400 Nuclear Magnetic Resonance Spectrometer operating at 400 MHz for proton and 75 MHz for carbon. Chemical shifts were recorded in ppm downfield of tetramethylsilane (TMS).

The article "Isolation, characterization and anti-inflammatory activity of compounds from the Vernonia amygdalina" was retracted in 2025. Reasons: unreliable results or conclusions; concerns about the citations; concerns about the authorship.

### 2.2 Preparation of Plant materials

The plant material (stem-bark and root) of *V. amygdalina* were harvested fresh from a botanical farm in Ilorin and authenticated by renowned taxonomist at the herbarium of the department of plant biology, University of Ilorin, Ilorin, Nigeria where the voucher (specimen) number UIL/001/972/2021 was documented.

### 2.3 Extraction, column chromatography Fractionation and isolation

The roots and stems were carefully rinsed with water to remove dirt and attached soil. The plant materials were shredded dried at ambient temperature without exposure to direct sunlight. They were blended into fine powder using electrical blender. The blended plant materials were extracted successively with solvents of increasing polarities separately. The mixtures was filtered and concentrated on a rotary evaporator (BUCHI) at reduced pressure. The extracts were stored in a refrigerator for further use. The methanol root and stem-bark extracts were dissolved in small amount of methanol and chromatographed independently over silica gel-loaded column using n-hexane, ethyl-acetate and methanol as eluting solvent system in polarity gradient order. 80 and 90 fractions were collected for the methanol root extract and methanol stem-bark extract respectively. Following TLC profiling, the fractions were combined to give 5 and 9 subfractions respectively. The subfractions obtained were subjected to another chromatographic elutions in a silica gel loaded column and some partially purified compounds that resulted were further purified via preparative thin layer chromatography or washing with selected solvents. Spectroscopic elucidation and comparison with literature data afforded three compounds which include luteolin-7-α-o-glucuronide (a flavonoid glycoside), vernoamyoside D (a triterpene glycoside), and vernotolaside (a bifuran glycoside).

### 2.4 *In vitro* albumin denaturing inhibition assay

The *in vitro* albumin denaturing inhibition assay was determined following standard protocol [23,24]. In order to obtain 2 mL reaction mixture, 1 mL 20 mM Tris HCl and 0.06 mg trypsin, buffered at pH 7.4 with the test samples (1 mL) of dilution range, 5–250 μg/mL was thoroughly mixed and incubated at 37 °C for 5 min before addition of 1 mL of prepared 0.8 % casein. The resultant mixture was inhibited for additional 20 min before 2 mL 70 % perchloric acid was adopted to terminate the reaction progress. The colloidal mixture that resulted was subjected to centrifugation and the absorbance taken at 210 nm while the buffer was adopted as blank. For each experiment, triplicate determination was made and the percentage inhibition was evaluated using the mathematical expression:

% Inhibition = 100 x (1 – V_s_/V_c_)

Where V_s_ = absorbance of test sample; Vc = absorbance of control.

The article "Isolation, characterization and anti-inflammatory activity of compounds from the Vernonia amygdalina" was retracted in 2025. Reasons: unreliable results or conclusions; concerns about the citations; concerns about the authorship.

### 2.5 Data analysis

IC_50_ - Half maximal inhibitory concentration, that is, the concentration that induced 50 % inhibition was estimated by using graphpad prism (software, inc, version 8.00), Nonlinear regression (curve fit), inhibitor against normalized response-variable slope. Significant difference of the mean of the replicate values was determined by the analysis of variance (ANOVA). Values at p < 0.05 were considered statistically significant.

## 3 Results and Discussion

The gravity column chromatography of the *V. amygdalina* methanol extracts afforded two known compounds from the root and a new compound from the stem bark. The structural elucidation of the compounds was based on the combination of data obtained from the proton and carbon-13 NMR Spectroscopy, Fourier Transform Infrared (FT-IR) Spectroscopy in comparison with literature data.

### 3.1 Infra-red spectra of crude extracts

The IR spectra data of the isolated compounds is as indicated in Table 1.

**Table 1:** FT-IR Spectra data of *V. amygdalina* column fractions.

Sample	*V*_O-H_ (cm^−1^)	*V*_C-O_ (cm^−1^)	*V*_C_=_O_ (cm^−1^)	*V*_C_=_C_ (cm^−1^)	*V*_C-H_ (cm^−1^)	*V*_CH__bend_ (cm^−1^)
Luteolin-7-α-o-glucuronide	3421	1271 1165	1710	1635	2922 2850	1377
Vernoamyoside D	3392	1263 1161	1718	1631	2937 2881	1384
Vernotolaside	3385	1263 1076		1635	2928	1411

### 3.2 IR spectrum of luteolin-7-α-o-glucuronide

The luteolin-7-α-o-glucuronide IR spectrum exhibited stretching vibration at 3421 cm^−1^ which underscore the presence of O–H stretch of alkanols while the C=O stretching at 1710 cm^−1^ was attributed to the presence of a saturated six-membered ring ketone. The C=C absorption band at 1521 cm^−1^ was alluded to that of non-conjugated alkane while the stretching vibration at 1635 cm^−1^ was attributed to conjugated double bonds. The C–H stretching at 2922/2850 cm^−1^ was characteristic of the aliphatic alkane while the C–O absorption band at 1271/1165 cm^−1^ indicated the presence of carboxylate. The FT-IR data obtained was in agreement with literature [25].

The article "Isolation, characterization and anti-inflammatory activity of compounds from the Vernonia amygdalina" was retracted in 2025. Reasons: unreliable results or conclusions; concerns about the citations; concerns about the authorship.

### 3.3 IR spectrum of vernoamyoside D

The IR spectrum of vernoamyoside D, which was compared with literature data [26] exhibited characteristic O–H stretching of alcohol at 3392 cm^−1^. The C=C absorption band appearing at 1631 cm^−1^ was attributed to the presence of conjugated alkene (Aromatic) while the vibration stretching at 1521 cm^−1^ was characteristic of an non-conjugated alkene. The C=O stretching at 1718 cm^−1^ was assigned to ketone group. The C–O stretch at 1263 cm^−1^ indicated the presence of carboxylic acid. The C–H stretch present at 2937 cm^−1^ confirmed the presence of an alkane C–H while the C–H bend of alkyl appeared at 1384 cm^−1^.

### 3.4 IR spectrum of vernotolaside

The IR spectrum of vernotolaside which was compared with some compounds in literature [26] confirms the presence of O–H of alcohol at 3385 cm^−1^ while the characteristic C–O stretching at 1263 cm^−1^ indicates the presence of carboxylate. The C=C absorption band at 1635 cm^−1^ corresponded to that of alkenes (aromatic) and the alkane C–H stretch was confirmed at 2928 cm^−1^. The C–H bend of alkene was exhibited at 1411 cm^−1^.

### 3.5 NMR data

The chemical shifts (δ) of the purified isolates, vernoamyoside D, luteolin-7-α-o-glucuronide, and vernotolaside obtained from methanol extract of *V. amygdalina* stem and root are depicted in Table 2.

**Table 2:** Chemical shifts (*δ*) of ^1^H/^13^C NMR of compounds isolated from *V. amygdalina*.

Luteolin-7-∝-o-glucuronide			Vernoamyoside D			Vernotolaside		
C/H Atom	^13^C (ppm)	^1^H (ppm)	C/H Atom	^13^C (ppm)	^1^H (ppm)	C/H Atom	^13^C (ppm)	^1^H (ppm)
2	171.1	___	1	35.2	1.2(d)	1	102.31	3.40
3	104.0	6.4(s)	2	28.3	2.4(d)	2	63.31	1.07
4	172.9	___	3	72.4	3.5(s)	3	82.08	____
5	160.2	8.1(s)	4	34.5	5.3(s)	4	97.16	____
6	99.5	6.2 (brs)	5	38.6	1.6(s)	5	60.66	2.42
7	170.2	___	6	29.7	3.4(d)	6	70.65	3.70
8	90.3	6.2 (brs)	7	57.3	7.3(s)	7	56.70	___
9	152.4	___	8	60.4	__	8	75.60	0.97
10	99.6	___	9	80.3	__	9	56.70	0.85
1^’^	120.2	___	10	62.4	__	10	78.42	3.68
2^’^	110.3	7.3(S)	11	40.3	3.4	sugar		
3^’^	145.6	8.2 (brs)	12	36.2	5.5(d)	1′	48.13	3.40
4^’^	150.0	7.4 (brs)	13	39.1	1.9(d)	2′	38.40	3.20
5^’^	115.9	6.8(s)	14	38.3	2.1(m)	3′	40.31	3.37
6^’^	119.2	7.4(s)	15	56.2	2.5	4′	36.76	3.10
Sugar			16	56.3	1.9	5′	39.50	3.38
1″	99.0	5.2(s)	17	44.2	1.4	6′	44.26	3.56
2″	70.0	5.1(s)	18	56.8	2.2	_	___	___
3″	72.0	5.3(s)	19	70.4	0.8(s)	_	___	___
4″	65.0	5.2(s)	20	76.4	0.6(s)	_	___	___
5″	63.0	5.2(s)	21	60.4	___	_	___	___
6″	nil	___	22	38.2	___	_	___	___
			23	45.1	7.4 (brs) _	_	___	___
_	_	___	24	50.4	5.2(m)	_	___	___
_	_	___	25	70.3	2.1(m)	_	___	___
_	_	___	26	40.4	0.8(d)	_	___	___
_	_	___	27	38.3	0.9(d)	_	___	___
_	_	___	28	29.4	___	_	___	___
_	_	___	29	44.0	2.0(s)	_	___	___
_	_	___	Sugar					
_	_	___	1′	74.5	4.1(d)	_	___	___
_	_	___	2′	79.0	2.8	_	___	___
_	_	___	3′	72.0	3.1	_	___	___
_	_	___	4′	77.3	3.0	_	___	___
_	_	___	5′	64.1	3.2	_	___	___
_	_	___	6′	58.3	3.4	_	___	___

**Luteolin-7-α-o-glucuronide**: Luteolin-7-α-o-glucuronide (Fig. 1) obtained as white powder was characterized using the infrared, proton and carbon-13 NMR data which were compared with the literatures [27]. The bands, 3392, 1718, 1631 and 1263 cm^−1^ corresponding to the O–H (Alcohol), C=O (carbonyl of esters), C=C_ar_ (conjugated alkene) and C–O (carboxylic acid) were confirmed. The carbonyl carbon at 171.1 ppm affirms the attribution. The compound was thus identified as luteolin 7-α-o-glucuronide (The glycone constituent was was established with the presence of the singlet protons at 5.2, 5.1, 5.3, 5.2, 5.2, 1.00 ppm and the prominent –OH proton signals resonating at 4.70–5.01 ppm). Luteolin-7-glucuronide is a known compound that has been confirmed in various medicinal plants and herbs. Its present has been confirmed in the aerial part *Antirrhinum majus* where it was confirmed to exhibit strong antimicrobial potential [28]. It has also been isolated in *Plantago lanceolata* [29], *Salvia ekimiana* Celep & Doğan [30], *Lycopus europaeus* L. [31], *Crataegus* x *macrocarpa* [32] and *Perilla frutescens* (L.) Britt [33].

The article "Isolation, characterization and anti-inflammatory activity of compounds from the Vernonia amygdalina" was retracted in 2025. Reasons: unreliable results or conclusions; concerns about the citations; concerns about the authorship.

**Fig. 1:** Structures of Vernoamyoside D, Luteolin-7- α-o-glucuronide and vernotolaside.

**Vernoamyoside D**: Following the extensive evaluation of the NMR data of the compound and in comparison with literature report [34], the structure (Fig. 1) was established without ambiguity. The glycosidic character of the compounds was affirmed by the proton and carbon signals at δ 5.45 and 74.5 respectively. This position was corroborated by the presence of the OH band at 3421 cm^−1^ in the infrared spectrum. Consequently, the identification of the compound as Vernoamyoside D was evidently aided by the combination of NMR data and the infrared report.

Vernoamyoside D, a stigmastane-type steroidal saponin has been isolated from the *V. amygdalina* of Chinese origin previously [34]. It was shown to possess varying degree of cytotoxicity on various cancer cell line. Vernonioside B₂ with vernoniamyoside A-D obtained from the leave of the plant alongside vernoamyoside D reportedly exhibited cytotoxicity on epithelial cells [34]. Other triterpenoids (stigmastane-type steroidal saponins; vernoamyosides and vernoniosides have been isolated from *Vernonia britteniana* also of the *Asteraceae* family. The compounds exhibited high *in vitro* cercaricidal activity with moderate *in vitro* antioxidant activities [35].

The article "Isolation, characterization and anti-inflammatory activity of compounds from the Vernonia amygdalina" was retracted in 2025. Reasons: unreliable results or conclusions; concerns about the citations; concerns about the authorship.

**Vernotolaside**: Vernotolaside, a quasi-new compound had structural similarity with bifuran glycoside. The NMR data (Table 2) structure was equivocal, as no additional 2D-NMR spectroscopic data was available. The total characterization will be done when the complete spectroscopic data are obtained.

### 3.6 *In vitro* albumin denaturing assay result

The *in vitro* albumin denaturation inhibition assay result for the crude extracts: VASAQ, VARAQ, VARMEOH, VASMEOH, VARNHEX, VASNHEX, VASETOAC and VARETOAC in comparison with diclofenac (control drug) are as presented, Table 3.

**Table 3:** *In vitro* anti-inflammatory (albumin denaturing potential) of crude extracts.

Conc (μg/mL)	VASAQ	VARAQ	VARMEOH	VASMEOH	VARNHEX	VASNHEX	VASETOAC	VARETOAC	Diclofenac
50	5.78 ± 4.31	10.69 ± 3.77	6.93 ± 2.75	10.11 ± 4.75	45.95 ± 4.16	43.64 ± 1.32	42.19 ± 1.52	37.57 ± 1.00	a32.37 ± 1.50
100	10.11 ± 5.62	12.13 ± 4.25	14.16 ± 2.64	17.63 ± 1.80	48.55 ± 4.07	48.84 ± 1.04	43.93 ± 1.04	43.64 ± 3.04	a37.86 ± 1.26
200	12.13 ± 6.37	14.16 ± 2.00	17.63 ± 2.18	20.52 ± 2.52	50.00 ± 4.19	48.26 ± 0.76	45.37 ± 1.32	46.24 ± 3.12	a44.50 ± 0.86
300	19.94 ± 4.81	17.91 ± 0.57	21.67 ± 1.60	22.83 ± 2.00	50.28 ± 3.62	50.86 ± 0.57	53.17 ± 1.32	44.79 ± 2.08	a52.60 ± 4.73
400	28.61 ± 1.60	19.94 ± 0.76	28.32 ± 0.76	25.14 ± 2.31	52.89 ± 3.21	54.62 ± 1.15	54.62 ± 4.62	51.15 ± 1.75	a64.74 ± 0.76
IC_50_ ± SEM	1092.00 ± 4.10	17729.00 ± 2.04	1614.00 ± 2.18	4378.00 ± 2.00	192.90 ± 4.19	195.50 ± 0.57	233.80 ± 1.34	446.30 ± 2.08	214.40 ± 0.88

Expressed data are mean ± standard error of mean of determinations made in triplicate.

VASAQ – *V. amygdalina* aqueous extract (stem), VARAQ – *V. amygdalina* aqueous extract (root), VARMEOH – *V. amygdalina* methanol extract (root), VASMEOH – *V. amygdalina* methanol extract (stem), VARAHEX – *V. amygdalina* n-hexane extract (root), VASEHEX – *V. amygdalina* n-hexane extract (stem), VASETOAC – *V. amygdalina* ethylacetate extract (stem), VARETOAC – *V. amygdalina* ethylacetate extract (root).

a - values at p < 0.05 are statistically significant.

The process by which external stimuli like heat, acid, base, organic chemicals, or inorganic salts trigger the protein to denature its tertiary and secondary structures is recognized as denaturation of protein [36,37] (Leelaprakash and Dass, 2011; SSen et al., 2015). Nonsteroidal anti-inflammatory drugs (NSAIDs) which acts as antigens has been used for the prevention of the protein denaturation [38]. However, the several side effects which included the induction of gastric irritation leading to gastric ulcers make the option less desired [39]. Hence, plant extracts or plant-derived compounds have reported some successes as protein denaturing inhibitions [40].

The article "Isolation, characterization and anti-inflammatory activity of compounds from the Vernonia amygdalina" was retracted in 2025. Reasons: unreliable results or conclusions; concerns about the citations; concerns about the authorship.

The VARNHEX and VASNHEX had higher albumin denaturing inhibition with IC_50_ at 192.9 and 195.5 μg/mL respectively than the polar extracts and the standard drug, diclofenac with IC_50_ 214.4 μg/mL. The strength of other extracts in the anti-inflammatory activity in decreasing order is thus: VASETOAC, VARETOAC, VASAQ, VARMEOH, VASMEOH and VARAQ. These activities were however lower when compared to VARNHEX, VASNHEX and diclofenac. Hence, VARNHEX and VASNHEX exhibited more potency as an anti-inflammatory substance.

The isolated compounds recorded moderate half-maximal inhibitory concentrations (IC_50_) thus: luteolin-7-α-o-glucuronide (379.5 μg/mL), vernoamyoside D (549.8 μg/mL) and vernotolaside (201.7 μg/mL) (Table 4). The IC_50_ values obtained were lower than that of diclofenac, 167.8 μg/mL. These compounds showed dose-dependent inhibition activities.

**Table 4:** Albumin denaturation inhibition potential of *V. amygdalina* isolated compounds.

Conc. (μg/mL)	Luteolin-7-α-o-glucuronide	Vernoamyoside D	Vernotolaside	Diclofenac
50	a10.19 ± 1.49	a17.84 ± 1.57	a34.56 ± 3.21	36.82 ± 0.56
100	a23.79 ± 1.49	a30.59 ± 1.49	45.60 ± 5.12	45.60 ± 0.98
200	a33.71 ± 0.84	a36.54 ± 1.41	a47.30 ± 3.89	52.97 ± 0.28
300	a47.02 ± 1.57	a41.07 ± 0.28	a55.24 ± 0.75	56.09 ± 1.13
400	a49.29 ± 1.13	a44.75 ± 1.47	a56.94 ± 0.28	57.50 ± 0.49
**IC**_**50**_**± SEM (μg/mL)**	**379.5 ± 1.49**	**549.8 ± 1.47**	**201.7 ± 3.89**	**167.8 ± 0.28**

Data are expressed as mean ± standard error of mean of triplicate determinations.

a - values at p < 0.05 are statistically significant.

The test samples showed significant dose-response albumin denaturation in the order; diclofenac, vernotolaside, luteolin-7-α-o-glucuronide and vernoamyoside D. The vernotolaside showed activity that is significantly comparable to the control, diclofenac. The result affirms that the *V. amygdalina* contain compounds with significant albumin denaturing inhibition potential. Plants are known to possess important bioactives with therapeutic potentials that are often useful for various applications particularly when preserved in appropriate form from the source [41]. Following the availability of essential minerals and bioactive compounds, folklores or plant-based formulations and decoctions are widely known for their ability to attenuate series of biological processes [[42], [43], [44]]. A polyherbal mixture containing *V. amygdalina* extract reportedly exhibited hepato and nephron-protective effect in animal model [45].

## 4 Conclusion

In this study, bioactive compounds with potential albumin denaturing inhibition potential were isolated using silica gel column chromatography from the *V. amygdalina* root and stem-bark. Utilising data from infrared, 1H, and 13C nuclear magnetic resonance spectroscopies as well as standard literatures, the characterization and structural elucidation of the purified compounds were achieved. The *in vitro* albumin denaturing inhibition was carried out on the extracts and isolated compounds using diclofenac as a standard. Three compounds which includes: luteolin-7-α-o-glucuronide, vernoamyoside D and vernotolaside were obtained. The compounds exhibited dose-dependent albumin denaturation inhibition with IC_50_ values of 549.8 μg/mL, 379.5 μg/mL and 201.7 μg/mL respectively. The vernotolaside would require further spectroscopic characterizations and *in vivo* biological evaluations. Apparently, *V. amygdalina* holds promise as a renewable source of bioactive natural products with prospective applications in the nutritional, pharmaceutical, and nutraceutical sectors. The findings of this study lend some credibility to the claim about the traditional application of the plant in alleviating issues associated with inflammation. However, further *in vivo* studies are required for the validation of the potentials of the isolated bioactives.

The article "Isolation, characterization and anti-inflammatory activity of compounds from the Vernonia amygdalina" was retracted in 2025. Reasons: unreliable results or conclusions; concerns about the citations; concerns about the authorship.

## Funding

This work was funded by Research Centre at King Fahad Medical City, Saudi Arabia through Grant number IRF#022-033.

## CRediT authorship contribution statement

**Olubunmi Atolani:** Writing – review & editing, Supervision, Software, Resources, Project administration, Methodology, Investigation, Funding acquisition, Formal analysis, Data curation, Conceptualization. **Mohammed Abubakar Usman:** Writing – original draft, Resources, Project administration, Methodology. **Jamiu Opeyemi Adejumo:** Methodology. **Adedamola Elizabeth Ayeni:** Resources, Methodology, Formal analysis. **Olamilekan Joseph Ibukun:** Validation, Formal analysis. **Adeola T. Kola-Mustapha:** Project administration, Funding acquisition. **Ngaitad S. Njinga:** Resources, Project administration, Funding acquisition. **Luqman A. Quadri:** Resources, Project administration, Funding acquisition. **Emmanuel O. Ajani:** Project administration, Funding acquisition. **Tajudeen O. Amusa:** Project administration, Funding acquisition. **Moji T. Bakare-Odunola:** Validation, Project administration, Funding acquisition. **Adenike T. Oladiji:** Resources, Project administration, Funding acquisition. **Athba Alqahtani:** Funding acquisition, Resources, Validation, Writing – review & editing. **Mohamed Abbas:** Funding acquisition, Resources, Visualization, Writing – review & editing. **Learnmore Kambizi:** Resources, Funding acquisition.

## Declaration of competing interest

The authors declare that they have no known competing financial interests or personal relationships that could have appeared to influence the work reported in this paper.
